The article "Privacy-Preserved In-Cabin Monitoring System for Autonomous Vehicles" was published in 2022. Journal: Comput Intell Neurosci.

# Privacy-Preserved In-Cabin Monitoring System for Autonomous Vehicles

**DOI:** 10.1155/2022/5389359

**Published:** 2022-04-22

**Authors:** Ashutosh Mishra, Jaekwang Cha, Shiho Kim

**Affiliations:** School of Integrated Technology, YICT, Yonsei University, Seoul, Republic of Korea

## Abstract

Fully autonomous vehicles (FAVs) lack monitoring inside the cabin. Therefore, an in-cabin monitoring system (IMS) is required for surveilling people causing irregular or abnormal situations. However, monitoring in the public domain allows disclosure of an individual's face, which goes against privacy preservation. Furthermore, there is a contrary demand for privacy in the IMS of AVs. Therefore, an intelligent IMS must simultaneously satisfy the contrary requirements of personal privacy protection and person identification during abnormal situations. In this study, we proposed a privacy-preserved IMS, which can reidentify anonymized virtual individual faces in an abnormal situation. This IMS includes a step for extracting facial features, which is accomplished by the edge device (onboard unit) of the AV. This device anonymizes an individual's facial identity before transmitting the video frames to a data server. We created different abnormal scenarios in the vehicle cabin. Further, we reidentified the involved person by using the anonymized virtual face and the reserved feature vectors extracted from the suspected individual. Overall, the proposed approach preserves personal privacy while maintaining security in surveillance systems, such as for in-cabin monitoring of FAVs.

## 1. Introduction

Intelligent monitoring and surveillance systems are widely used to ensure safety and security. Popular applications of monitoring in public are video surveillance cameras (closed-circuit television); monitoring in intelligent transportation systems, including in-cabin monitoring and road traffic monitoring; and video monitoring for data generation and navigational tasks around city centers, airports, and public roads [1]. Driving automation also requires public visual information for multiple tasks [2]. The Society of Automotive Engineers defined six levels of autonomy in driving automation in 2014 (from no automation (level 0) to full automation (level 5)) [2–4]. Level 4 autonomous vehicles (AVs) are highly automated and capable of performing all driving tasks under certain conditions without human intervention. However, the driver (human) may control such AVs as and when required. In particular, fully autonomous vehicles (FAVs) (level 5 AVs) have no drivers; all occupants are passengers only [3, 4]. Therefore, no one oversees such AVs. In addition, in public and shared vehicles (such as ridesharing, carsharing, and car-full services in AVs), the passengers do not know each other. Therefore, it is important to ensure the security and safety of all occupants sitting in the cabin of such AVs. Furthermore, the vehicle should be protected from any malicious behavior of the occupants and/or external threats. Therefore, FAVs essentially require a multipronged in-cabin monitoring task in real time [5]. However, many countries have imposed a ban or severe restrictions on facial recognition techniques to secure personal information [6–16]. There are legal and ethical issues that impose various restrictions on public monitoring and surveillance systems [16–19]. Furthermore, identification of the accused is also important in abnormal (irregular) situations. This study was motivated by the fact that facial monitoring is important for safety; however, it poses a threat to individual privacy. In this study, we focused on the following two problems associated with in-cabin monitoring systems (IMSes):

- Protection of facial privacy.
- Evidence of the accused in abnormal situations.

The article "Privacy-Preserved In-Cabin Monitoring System for Autonomous Vehicles" was published in 2022. Journal: Comput Intell Neurosci.

Therefore, a robust solution is required to provide privacy-preserved monitoring in public [20]. Moreover, it should be capable of identifying the concerned person when required.  Figure 1 shows the dilemma of intelligent monitoring systems.

As illustrated in the above figure, an anonymous face protects personal information during in-cabin monitoring of an FAV. However, in certain irregular situations, personal identity is required to identify the accused person. An example of an abnormal incident or irregular situation can be an occupant of the FAV acting violently or attempting vandalism against the other occupants or toward the FAV itself. In such cases, it is important to identify the concerned person. Furthermore, this is an abnormal situation; however, in-cabin monitoring with real faces is not a solution to this problem. The breach of facial information leads to multiple consequences, such as misuse of facial data and banking and financial fraud [1, 6, 7, 13, 14]. One of our motivations for this work was to provide an approach that can protect against such problems in public monitoring systems, particularly the IMS. In-cabin monitoring with facial anonymization has security issues, while those with facial identity have privacy issues. Therefore, it creates a contradiction between privacy and security.

### 1.1. In-Cabin Monitoring

In-cabin monitoring is important in level 4 and beyond AVs [5]. It provides safety and security to the occupants. Simultaneously, it provides safety to the vehicle itself in an irregular situation. Past research works include in-cabin monitoring in various situations [21]. In-cabin monitoring for violence detection inside a FAV was reviewed in [22]. Bell et al. performed in-cabin monitoring to detect harsh vehicle maneuvers and risky driving behaviors [23]. Szawarski et al. patented the idea of in-cabin monitoring for a monitoring vehicle seat, occupants inside a vehicle, and the orientation of both the occupants and the vehicle seat [24]. Safety and cleaning problems of in-cabin monitoring of a vehicle were presented in [25]. However, a monitoring system should protect against any breach of personal privacy (facial identity) with the simultaneous ability to identify an actual person in case of irregular situations.

The article "Privacy-Preserved In-Cabin Monitoring System for Autonomous Vehicles" was published in 2022. Journal: Comput Intell Neurosci.

### 1.2. Facial Privacy versus Facial Recognition in Monitoring Applications

Real-time monitoring is essential in multiple monitoring applications. However, privacy in the public domain is an important concern in real-time monitoring tasks [26–30]. Facial anonymization is a common practice for preserving personal privacy. Recently, generative adversarial network- (GAN-) based deep learning (DL) models have been widely used for face swapping and anonymization [31–34]. In our previous study [31], we demonstrated a robust approach to preserving the facial identity of the occupants in a FAV cabin. It incorporated the facial swapping and reenactment technique to maintain privacy in in-cabin monitoring. However, in ab abnormal situation, the anonymized face of the occupants made it difficult to identify the concerned person [20].

### 1.3. Our Key Research Highlights

In this study, we propose an intelligent IMS. It is an efficient approach for identifying a person, even with an anonymized face. This method resolves both privacy and security issues. Accordingly, we can identify the person who causes an irregular situation, even with their anonymized face. In this approach, we preserved the key facial information of the occupants and stored these identity features on the cloud. These key features help in recognition of the person involved in the irregular situation. The highlights of this study are as follows:

- The concept of having an appropriate source face for each target face enhances puppeteering and reenactment of facial emotion and behavior. It helps in event and behavior detection in intelligent monitoring and surveillance systems in the public domain.
- The involvement of the two-dimensional (2D) landmark position in the reenactment generator and separate segmentations of face and hair in the segmentation generator with inpainting and blending generators enhances the facial anonymization and reenactment operations.
- The 128D identity feature is a key marker for accurate facial identification in an anonymized domain. The concept of storing a pair of IDs (original and anonymized) leads to reidentification without any privacy threat. It is not possible to know the original face with only 128D identity features. For reidentification, both the original visual input and the ID are required. In the cloud, the anonymized visual image with the original *ID* is stored. Therefore, there is no threat of privacy breach, even though the *IDs* are stored in the cloud.
- Therefore, the proposed approach augments the facial identity feature information to locate the involved person in any abnormal situation without any personal privacy breach.

The article "Privacy-Preserved In-Cabin Monitoring System for Autonomous Vehicles" was published in 2022. Journal: Comput Intell Neurosci.

This approach pioneers a newer method of monitoring and surveillance to avoid any legal or ethical issues. Therefore, a monitoring database can be created in the anonymized domain, thereby facilitating further research on events and behavior monitoring in the public domain.

## 2. Materials and Methods

Personal privacy with identification is a challenge as well as a demand in real-time monitoring applications [20]. In this study, we developed a privacy-preserved IMS with the reidentification capability that can identify the accused person. The framework of the proposed method is shown in Figure 2. The proposed system operates in three stages. In stage 1, facial anonymization was performed to ensure personal privacy. It was performed using the onboard device of the AV. In stage 2, a pair of identity features (*ID*s) was generated for each face before and after anonymization (*ID*_*R*_ and *ID*_*A*_). Further, the anonymized video along with the *IDs* was fed to the cloud. The pairs of *IDs* were kept in the cloud for person reidentification when required. The anonymized video frames were sent to the data center for further processing (monitoring and surveillance). In stage 3, the *IDs* were matched to search the accused (person involved in an irregular situation (*ID*_*A_AS*_)). During the investigation, the similarity between *ID*s ensured the identification of the concerned person (*ID*). Further, during the investigation, this approach was verified by matching the *IDs* of the suspect face (*ID*_*inv*_) at the time of investigation with the accused person's *ID*.

The dilemma between monitoring requirements and legal and ethical issues is also resolved through this approach. The details of the proposed approach are discussed thoroughly in Section 2.2. This approach is suitable for creating a monitoring and surveillance database with legitimation.

### 2.1. Materials

Many research works have been published on personal privacy and person identification considering these two issues as separate research problems. In this study, we briefly surveyed the related works and developments on both face anonymization and person identification.

The article "Privacy-Preserved In-Cabin Monitoring System for Autonomous Vehicles" was published in 2022. Journal: Comput Intell Neurosci.

#### 2.1.1. Face Anonymization

Face deidentification preserves privacy-sensitive information. It alters the original face to hide privacy-sensitive information. Anonymization of faces is an easier and more robust solution to personal privacy-related threats in the digital domain [35]. Blurring, masking faces, or creating a patch over faces is slightly easier than any other face anonymization approach; however, those methods suffer from significant loss of facial information [32, 36]. Therefore, face swapping has attracted significant attention for facial anonymization purposes. The morphable model-based facial exchange approach is considered a pioneering work in face swapping [37]. Bitouk et al. demonstrated automatic face replacement in their work [38]. Machine-learning-based face swapping was suggested in [39]. A convolutional neural network (CNN) was used for face segmentation and swapping in [40]. GAN-based deep models have become popular for virtual human face generation [33, 34]. Therefore, along with autoencoders, GAN-based face swapping has gained considerable attention among researchers for seamless end-to-end face anonymization [33, 34, 41]. Face swapping-based automatic generation and editing of faces was showcased in [42]. It used a region-separative GAN (RSGAN). An autoencoder-based algorithm for face swapping was presented to detect fake videos [43]. In [44], a GAN-based encoder-decoder network was suggested to swap human faces. Collateral privacy issues have also been resolved using the face swapping method [45]. Nirkin et al. suggested a face swapping GAN (FSGAN) in [46]. It provided subject agnostic face swapping and reenactment between a pair of faces. Naruniec et al. presented a fully automatic neural face swapping method in [47]. Sun et al. proposed a hybrid model for face anonymization [36]. Hukkelas et al. introduced a GAN-based DeepPrivacy architecture for face deidentification to remove all privacy-sensitive information [34].

#### 2.1.2. Person Identification

Facial recognition has multipurpose objectives, such as recognition, classification, and discrimination. Urbanization and smart cities demand widespread applications for face recognition [48–52]. Therefore, various face recognition approaches involving person identification have been demonstrated by past researchers. Face recognition approaches are classified into three categories: local, holistic, and hybrid approaches [52]. Local approaches involve only partial facial features (such as eyes, mouth, and nose) to recognize a face, whereas holistic approaches involve complete facial features, including background for facial recognition. Hybrid approaches, as the name suggests, involve both local and holistic approaches. In holistic approaches, popular algorithms involve independent component analysis, linear discriminative analysis, and principal component analysis [53, 54]. The development of artificial intelligence (AI) incorporating DL and CNNs has boosted the performance of facial recognition algorithms. Taigman et al. presented a deep neural network-based face recognition system, *DeepFace* [55]. Furthermore, many other extended versions of *DeepFace* have been demonstrated in multiple studies [56–59]. Adjabi et al. thoroughly reviewed face recognition techniques and their comparisons and future scope in their study [51]. Kortli et al. surveyed popular face recognition techniques in all three categories, that is, local, holistic, and hybrid approaches, in their study [52]. They compared these techniques in terms of accuracy, complexity, and robustness. They also discussed the advantages and disadvantages of the respective approaches. Wang et al. efficiently surveyed DL-based face recognition techniques in their study [60]. They exhaustively reviewed various popular DL-based approaches, including autoencoder-based, CNN-based, and GAN-based techniques. They also enumerated the key features, advantages, and disadvantages of these techniques. Furthermore, they summarized some of the commonly used datasets for deep face recognition. Moreover, they indexed the emerging real-world issues and major technical key challenges in deep facial recognition.

The article "Privacy-Preserved In-Cabin Monitoring System for Autonomous Vehicles" was published in 2022. Journal: Comput Intell Neurosci.

However, an application involving person identification must address important privacy concerns [61]. In particular, facial identification in the public domain must tackle individual freedom and ethics-related issues [51, 62]. Therefore, the state-of-the-art research problem in face recognition is the reidentification of an individual on anonymized data. Rocher et al. demonstrated the likelihood of correctly reidentifying a specific individual, even with the anonymized dataset [30]. They suggested a generative graphical model that can be trained on incomplete data to accurately identify individuals. Rooijen et al. suggested 2D video tracking for the reidentification of individuals in an anonymized dataset [20]. They suggested that the real facial information of a person is not necessary for reidentification. Luo et al. suggested effective training tricks for person reidentification [63]. A residual learning framework using the residual network (*ResNet*) model was suggested in [64] for visual recognition tasks. This facilitated the easier and more efficient training of a substantially deeper network. Schroff et al. suggested unified embedding using only 128 bytes per face for efficient face recognition [65]. They developed their network by incorporating the batch input layer and deep CNN, followed by normalization. They used triplet loss to minimize the training errors. The world's simplest face recognition library (Dlib face recognition) is a popular and efficient tool for extracting facial landmarks [66]. It is a cross-platform open-source machine-learning toolkit that supports the development of machine-learning algorithms. It helps in recognizing and manipulating faces. Intent and behavior have been successfully detected using various techniques. Facial gesture sensing is performed using virtual reality (VR) and augmented reality (AR) devices, respectively in [67, 68]. AR/VR devices provide sensor responses to detect the intent or behavior of the user. However, FAV in-cabin monitoring requires intent or behavior detection using visual (computer vision (CV)-based) monitoring approaches.

The article "Privacy-Preserved In-Cabin Monitoring System for Autonomous Vehicles" was published in 2022. Journal: Comput Intell Neurosci.

### 2.2. Method

In this study, we proposed a representation learning-based approach to generate the identity signature of occupants. This signature is capable of deidentifying a person concerned with an irregular situation in the cabin of level 4 and beyond AVs. We proposed facial anonymization and reidentification system to provide countermeasures in case of an irregular situation. Therefore, this method provides personal information security with traces of the concerned person in case of any abnormality. The proposed method includes four main tasks. First, face anonymization with reenrollment. This is performed by using the face agnostic face swapping technique. It uses a set of GANs. These GANs are used for three purposes: facial reenactment and segmentation, facial inpainting, and facial blending. After accomplishing face anonymization, the second task is to extract the facial identity features of the occupant's faces in pairs (before and after anonymization, i.e., *ID*_*R*_ and *ID*_*A*_) using the *ResNet*-based model. These *IDs* are stored in the cloud, and the anonymized video frames of in-cabin monitoring are transferred to the data center via the cloud for further processing. The third task of the proposed approach is to identify the accused by identity feature matching. Similarity matching of the *ID* of the accused obtained at the data center with the *IDs* of the occupants stored in the cloud ensures the identification of the concerned person (*ID*_*A*_). However, it is the *ID* of the anonymized face of the accused. The Euclidean distance metric was used for similarity matching. Similarly, using the stored pairs of *IDs* (IDR and *ID*_*A*_), we can obtain the real face identity feature of the accused (*ID*_*R*_). Finally, in the fourth task, the evidence of the accused is obtained by matching the similarities between the *IDs* of the suspects with the *ID* of the accused during an investigation. Further details of the proposed method are provided in the following sections.

The article "Privacy-Preserved In-Cabin Monitoring System for Autonomous Vehicles" was published in 2022. Journal: Comput Intell Neurosci.

#### 2.2.1. Facial Identity Feature Vector

The facial identity feature is (128, 1)-dimensional encoding of a facial image. It contains the encoded landmarks of the face using the *ResNet* model. The FaceNet-based CNN model and Facedlib face recognition library are used to extract the 128D identity features (*ID*) from the faces. Additionally, 128D is optimal embedding, which results in appropriate features required for reidentification or measuring the similarity between two faces. It has already been validated in the “*FaceNet*” architecture that fewer than 128D identity features deteriorate the identification performance; however, increasing the dimension only unnecessarily increases the number of parameters. This is the main reason for adopting the 128D identity features for recognizing faces.

Figure 3 shows the (128, 1)-dimensional facial identity feature vector generation of the occupant's face image. It uses a *ResNet*-based architecture consisting of 29 convolutional layers for this purpose. The *ResNet* architecture facilitates the dipper layer accessibility. Additionally, they have an inherent tendency to minimize the training error loss by increasing the number of layers. The triplet loss function is used to estimate the error in the reidentification of the concerned person. It performs similarity matching on the 128D identity features. For the anonymized anchor image *ID* (*I*_*A*_), positive anonymized image *ID* (*I*_*P*_), and negative anonymized image *ID* (*I*_*N*_), the triplet loss is estimated by the following equation:

(1) $$\begin{array}{c} ℒ\left(A,P,N\right)=\max\left(\|I_{A},I_{P2}\|-\|I_{A},I_{N\|2}+\mathrm{margin},0\right). \end{array}$$

The anonymized anchor image ID (IA) represents the 128D ID of the person figured out in an irregular situation. The positive anonymized image (IA) is the stored image 128D ID of the same person on the cloud, and the negative anonymized image ID (IA) is the 128D ID of another occupant. Here, (‖x, y‖_2_) denotes the “Euclidean distance” between pairs {*x*, *y*} in the triplet loss function. A factor margin is included in equation (1) to reduce the chances of misclassification. These facial features are incorporated in 128D encoding and are used as the facial recognizer using only 128 bytes per face.

The article "Privacy-Preserved In-Cabin Monitoring System for Autonomous Vehicles" was published in 2022. Journal: Comput Intell Neurosci.

Furthermore, a distance-based classifier compares the 128D features to identify the person involved in an irregular situation. It represents the difference between two feature vectors in Euclidean space. Suppose that image (*R*) represents the person. Image (*C*) is the stored image (copy) of the same person on the cloud, and image (*D*) is an image of another occupant. Further, *ƒ*(*x*) represents the 128D encoding of the image *f*(*x*). The similarity (*S*) in the vector space is measured by the following equation:

(2) $$\begin{array}{c} S=\text{min}\left(\|f\left(R\right),f{\left(C\right)\|}_{2},\left(\|f\left(R\right),f{\left(D\right)\|}_{2}\right)\right). \end{array}$$

It guarantees that images (*R*) and (*C*) are of the same occupant and are different from image (*D*), which is the image of another occupant.

#### 2.2.2. Source Image Generation

A source image was required for face swapping in facial anonymization. It is used to replace the face appearing in the target image. This replacement, that is, swapping, should produce a realistic result that seamlessly reenacts the anonymized face that is similar to the target face. Our recommendation is to use a nonreal face as the source image. It mitigates any chaos/conflicts that may occur by using any real face as the source image. Therefore, in our proposed method, we used GAN-generated virtual human faces as the source image. We have considered generating appropriate source faces that can effectively render the original emotions or behaviors performed by the occupants. It helps in further event and behavior-monitoring tasks.  Figure 4 shows the proposed source image generation process. We applied the concept of similarity matching in vector space to select a similar source face for each target face from the set of virtual human faces (nonreal face as the source image). Similarity matching between source and target faces facilitates reciprocating similar emotions and intents, which is necessary for further monitoring applications.

Figure 4 shows the source image generation process. The face detector detects the faces (target faces) of the occupants (from the in-cabin visual input). The identity feature extractor extracts the *IDs* (128D identity features) of faces (target faces) and matches the similarity of the target faces with the set of virtual human faces (source faces) to find the most appropriate source face. This similarity matching is in the vector space (Euclidean distance matching between the extracted face *ID* and *IDs* of the set of virtual human faces).

#### 2.2.3. Facial Anonymization

Facial anonymization requires exactitude in the anonymized faces to mitigate errors in further processing. Therefore, swapping should be performed efficiently to provide unaltered expressions and emotions over the anonymized face. We used the concept of FSGAN for facial anonymization to provide personal privacy during in-cabin monitoring of irregular situations. This requires perfection in the following three tasks:

*(i) Facial Reenactment and Segmentation*. To obtain proper facial swapping, we must estimate the proper reenacted face. This is performed by the proper segmentation of the face and hair segments of the target image. Proper facial reenactment requires separate face and hair segmentations with the mapping of 2D facial landmark positions. Therefore, the stepwise loss function is considered as the objective function for implementing facial reenactment. For *i*^th^ layer feature map (*F*_*i*_ ∈ ℝ^*C*_*i*_×*H*_*i*_×*W*_*i*_^), the perceptual loss (ℒ_perc_) between pairs of images (*x*, *y*) is expressed as follows:

(3) $$\begin{array}{c} {ℒ}_{\text{perc}}\left(x,y\right)=\sum \frac{1}{C_{i}\times H_{i}\times W_{i}}\;\times \|F_{i}\left(x\right),F_{i}{\left(y\right)\|}_{2}\text{.} \end{array}$$

The reconstruction loss (ℒ_rec_) between a pair of images (*x*, *y*) is expressed as follows:

(4) $$\begin{array}{c} {ℒ}_{\text{rec}}\left(x,y\right)=\lambda_{\text{perc}}\times {ℒ}_{\text{perc}}\left(x,y\right)+\lambda_{\text{pixel}}\times {ℒ}_{\text{pixel}}\left(x,y\right), \end{array}$$

where “*λ*” is the corresponding hyperparameter (*λ*_perc_=1; *λ*_pixel_=0.1; *λ*_adv_=0.001; *λ*_*SG*_=0.1; *λ*_rec_=1; *λ*_stepwise_=1) and *λ*_reenactment_ is linearly increased from 0 to 1 during training. Pixelwise loss (ℒ_pixel_) between a pair of images (*x*, *y*) is calculated as (ℒ_pixel_(*x*, *y*)=*‖x* − *y‖*). We have used the multiscale discriminator adversarial loss objective function to improve the realism of the generated images. The adversarial loss (ℒ_adv_) between the generator and discriminator (*G*, *D*) is expressed as follows:

(5) $$\begin{array}{c} {ℒ}_{\text{adv}}\left(G,D\right)=\min\left(\max\left(\sum {ℒ}_{\text{GAN}}\left(G,D\right)\right)\right),\\ {ℒ}_{\text{GAN}}\left(G,D\right)=E_{\left(x,y\right)}\left[\log\;D\left(x,y\right)\right]+E\left(x\right)\left[\log\left(1-D\left(x,G\left(x\right)\right)\right)\right], \end{array}$$

where “*E*_(*x*, *y*)_” is the expected value over all real data instances. “*E*_(*x*)_” is the expected value over all random inputs to the generator. The reenactment generator loss (ℒ_*RG*_) is given by the following equation:

(6) $$\begin{array}{c} {ℒ}_{RG}={ℒ}_{\text{perc}}+{ℒ}_{\text{rec}}+{ℒ}_{\text{adv}}. \end{array}$$

The perpetual loss is used to estimate the errors in capturing fine facial details, and the reconstruction loss is used to evaluate pixelwise color inaccuracy. Adversarial loss improves the generated images and provides a realistic look. The standard cross-entropy loss (ℒ_*CE*_) is defined as (for truth label “*t*_*i*_” and the “*SoftMax*” probability “*P*_*i*_” for *i*^th^ class)

(7) $$\begin{array}{c} {ℒ}_{CE}=-\sum t_{i}\times \;\log\left(P_{i}\right). \end{array}$$

Further, segmentation generator loss (ℒ_*SG*_) is obtained by the following equation:

(8) $$\begin{array}{c} {ℒ}_{SG}={ℒ}_{CE}+{ℒ}_{\text{pixel}}. \end{array}$$

*(ii) Facial Inpainting.* This method estimates the missing portions of the reenacted face based on the face and hair segmentation of the target image. The inpainting generator loss (ℒ_*IP*_) was calculated using the following equation:

(9) $$\begin{array}{c} {ℒ}_{IP}={ℒ}_{\text{rec}}+{ℒ}_{\text{adv}}. \end{array}$$

(iii) *Facial Blending*. It blends the completely reenacted face such that the swapped face matches the background environment like the original target face. The loss function (ℒ_*B*_) for facial blending is obtained using the following equation:
  (10) $$\begin{array}{c} {ℒ}_{B}={ℒ}_{\text{perc}}+{ℒ}_{\text{adv}}. \end{array}$$

The identity signature is generated corresponding to each occupant (a pair of identity signatures for real and anonymized faces) in the FAV. After facial anonymization, the video frames are transmitted to the cloud along with a pair of identity signatures of the occupants.

The article "Privacy-Preserved In-Cabin Monitoring System for Autonomous Vehicles" was published in 2022. Journal: Comput Intell Neurosci.

#### 2.2.4. Anonymized Person Reidentification in Abnormal Situations

The proposed IMS facilitates the reidentification of the person involved in an abnormal situation. In our algorithm, in-cabin facial anonymization for preserving identity before transmitting the video frames to the cloud was achieved through the following pseudocode. The identity signature is generated corresponding to each occupant in the FAV. It is a vector of size 1 × 128. Therefore, for each occupant, we have a pair of identity signatures corresponding to the original and anonymized faces. Each pair is stored in the cloud. In any irregular situation, the concerned person is back-traced by matching the identity signature and anonymized face. The following is Pseudocode 1 of our proposed approach for obtaining the identity features (*ID*) of the person involved in an abnormal situation.

We considered virtual human face generation for the source faces. These faces are used to swap the target face in the captured visual in-cabin dataset. The source faces are generated depending on the similarity of the target face in the vector space. A similar source face provides the exactitude in replaying the facial gestures. This facilitates better reenactment performances. The concept of virtual human face generation for the source face protects any chaos or risk of threatening others' identities. Furthermore, we generated the facial identity signatures of the original and anonymized faces. These identity signatures help backtrack the concerned person in the event of an irregular situation. The identity signature is only vectored information. In other words, the identity signature in our proposed approach is extracted from a face that is used to reidentify the face. However, a face cannot be recreated using this information. Therefore, personal identity is not revealed through the identity signature. Our proposed approach provides proof or evidence that confirms the identity of the concerned person. The following is Pseudocode 2 of our proposed approach for evidence of the person involved in an abnormal situation.

The article "Privacy-Preserved In-Cabin Monitoring System for Autonomous Vehicles" was published in 2022. Journal: Comput Intell Neurosci.

In the case of proof or evidence, our method determines who is the concerned person. The returned identity feature (real face *ID*_*R*_(*k*)) in Pseudocode 1 refers to the crucial identity parameter of the person involved in an abnormal situation. Matching the identity feature at the time of investigation with the obtained *ID* (real face *ID*_*R*_(*k*)) confirms the person involved in an abnormal situation. Therefore, this approach easily locates the person involved in an irregular situation without any breach of others' identities.

## 3. Results and Discussion

In our experiment, we first anonymized the occupants of the FAV to secure their privacy in the public domain. Further, we applied the concept of vector space similarity to match the representation learning-based identity features for face recognition to locate the person involved in an irregular situation. The augmentation of the representation-learning-based identity feature introduces a new domain in reidentification. The proposed system was introduced to maintain personal privacy during the monitoring. We examined our proposed system for the in-cabin monitoring task of the FAV. We captured our database for in-cabin monitoring in abnormal situations. The similarity measure (*S*_*i*,*j*_) is calculated by the Euclidean distance (ED) metric that is expressed as follows:

(11) $$\begin{array}{c} S_{i,j}=\|f\left(i\right),f{\left(j\right)\|}_{2}, \end{array}$$

where ƒ(*i*) and ƒ(*j*) represent the 128D encoding of images *i* and *j*, respectively. Therefore, the similarity measure identifies the distance (Euclidean distance) between two pairs of *IDs* (128D encoding). The lesser the distance is, the closer the faces are.

### 3.1. Appropriate Source Faces

We proposed the concept of an appropriate source face in our facial anonymization approach. For every occupant face (target face), an appropriate source face is obtained by matching their similarity in the vector space. We considered various scenarios to assess the efficacy of our proposed approach, including single and multiple faces in the input image frame.  Figure 5 shows the complete set of the considered source faces in our experiment. We considered a set of 24 source faces (shown below). All these faces were not real (AI-generated). The source faces were used to swap the target face in the facial anonymization process.

The article "Privacy-Preserved In-Cabin Monitoring System for Autonomous Vehicles" was published in 2022. Journal: Comput Intell Neurosci.

These faces are nonreal virtual human faces. Generated Photos provides GAN-generated faces, which are human faces of nonreal humans. This has the benefit of further augmentation in anonymization. We considered various scenarios in our experiments. Examples include images with a single face only (for both males and females), multiple faces for males only and females only, and multiple faces for both males and females. These are in-cabin images obtained from the public domain (through an image search on the web) and are shown in Figure 6. We considered different scenarios for the occupants in the cabin. Therefore, in F1 and F2, there is only a single person in-cabin (F1: male and F2: female). In other scenarios, we considered more than one person in the cabin (only males, only females, and both males and females). Finally, we considered a family with children. There are four most appropriate source faces (S1 to S4) chosen for face anonymization.

Table 1 presents the similarities (in vector space) between the source and target faces, as shown in Figures 5 and 6.

These values follow the facial similarities of the source and target faces. These values measure the distance between the identity features of the source and target faces. The lower the values are, the more similar the faces are. The values in the green boxes represent the minimum Euclidean distances. These minimum values indicate appropriate source faces for anonymization. We can observe that the male target faces have lesser distances for male source faces than for female source faces. Interestingly, the distance values follow the similarity in looks as well. The eastern looks target faces have a lesser distance for eastern source faces than for the western source face, and vice versa. Female source faces have a lesser distance than the identity features of children's target faces.

### 3.2. Privacy Preservation during In-Cabin Monitoring

Facial anonymization is performed after deciding the appropriate source face using FSGAN-based face swapping and reenactment.  Figure 7 depicts the reenacted anonymization of the target faces. Here, the first row (F1 to F8) and the third row (F9 to F23) show the original in-cabin visual inputs, and the corresponding anonymized output is represented in the second row (A1–A8) and fourth row (A9–A23). We chose four source faces (S1 to S4 shown in Figure 6) to swap the target faces (F1 to F23).

The article "Privacy-Preserved In-Cabin Monitoring System for Autonomous Vehicles" was published in 2022. Journal: Comput Intell Neurosci.

It is evident from this result that perfect reenactments are achieved even in the anonymized domain. Thus, it discerns the preservation of personal privacy during monitoring and surveillance operations. Furthermore, this appropriate reenactment supports the detection of abnormal or irregular situations in real time. To examine abnormality detection in the anonymized domain, we have experimented by considering vandalism as an irregular situation inside the vehicle cabin. We created our database for a similar situation. Snippets of the vandalism inside the vehicle are shown in Figure 8. We created a situation wherein occupants in the back seat of the vehicle started fighting with the occupants in the front seat. Four scenes were captured in our experiment. Shoulder shaking is shown in scene #1. Scene #2 shows a slapping scenario. Head shaking is discerned in scene #3, and scene #4 represents a neck choking incident inside the cabin of the vehicle. The identity features (*ID*s) of each occupant were calculated for normal and irregular situations. It is clearly observed that O3 (in the green box) is responsible for the irregular situation (in-cabin vandalism of the vehicle shown in the red box).

### 3.3. Person Reidentification in Abnormal Situations

Table 2 presents the similarities of the anonymized identity feature (*ID*_*A*_) with the anonymized facial identity feature of occupant #3 (*ID*_*A_IS*_). Here, *ID*_*A_IS*_ is the anonymized identity feature of the occupant who is involved in an irregular situation calculated at the data center, and *ID*_*A*_ is the anonymized identity feature of the occupant stored in the cloud.

The values in the green boxes represent the minimum Euclidean distances. These minimum differences between the *ID*s indicate the involved person. The original *ID* of this person is stored in the cloud. Therefore, by mapping the *ID*, we can easily identify the real person. Reidentification was performed by backtracking the *ID* obtained from the cloud and pictures of the occupants taken during the investigation. The *ID* of the person involved in an abnormal situation from the cloud (*ID*_*R*_) needs to be matched with the *ID*s of the occupants inside the vehicle for facial identification of the person. This approach provides proof or evidence confirming the identity of the concerned person. For assurance of the person involved in the abnormal situation, we took pictures of the occupants (during an investigation). The images are shown in Figure 9. Now, the identity feature of each occupant is extracted to match the concerned person *ID* (*ID*_*R*_) (as per Pseudocode 2). First, we compared the similarity between the faces of the occupants inside the vehicle with those of the other faces captured during the investigation. This is required to ensure that the occupants are the same.

The article "Privacy-Preserved In-Cabin Monitoring System for Autonomous Vehicles" was published in 2022. Journal: Comput Intell Neurosci.

Table 3 presents the similarity measures between the occupants' *ID*s extracted during an investigation and their *ID*s extracted from the in-cabin images.

The minimum Euclidean distances are represented by the green boxes. Here, minima indicate that the occupants O and O′' are the same. Thereafter, assurance of the involved person is performed by matching the identity feature of the occupants extracted from the in-cabin image of the vehicle with the *ID* of the person involved in an abnormal situation (stored in cloud *ID*_*R*_).  Table 4 presents the similarity measures between the occupants' *ID*s extracted from the in-cabin image with the obtained *ID* of the person involved in an abnormal situation (stored in cloud *ID*_*R*_).

The zero value in the green box indicates that the occupant (O3) is the person involved in an abnormal situation. Overall, this approach focuses on in-cabin monitoring with personal privacy preservation to avoid abnormal situations. Personal privacy preservation is achieved by using the concept of event and behavior monitoring in an anonymized domain. The person's reidentification is only for providing evidence in cases where the involved person is denying it.

## 4. Conclusions

Identity feature augmentation in anonymization is a potential solution for providing privacy in public domain monitoring. Identification of the involved person is crucial, especially in abnormal situations. The proposed intelligent IMS augments the security features with privacy. This method is suitable for creating a monitoring database without any restrictions or legalities. We performed various scenarios to assess the efficacy of the proposed system. It provided an efficient algorithm to perform monitoring tasks in the public domain without any threat to the personal identity of a person. This helped in reidentification, even with an anonymized face. In the future, this algorithm can be implemented on various public domain monitoring platforms, such as transportation systems, shopping centers, theaters, hospitals, highways, fuel refilling stations, smart city applications, and toll plazas.

## Figures and Tables

**Figure 1:** System overview of the proposed IMS. (a) Few examples causing abnormal situations in the cabin of a vehicle. (b) The dilemma of the legal and ethical issues (privacy) and practical problems (requirement of monitoring). Case 1: the masked face has no facial information, which is crucial in surveillance and monitoring inside the cabin of a vehicle. Case 2: real face suffers from personal privacy threats. Case 3: facial anonymization solves the problem of privacy; however, it has the problem of identifying the concerned person in case of irregular situations.

The article "Privacy-Preserved In-Cabin Monitoring System for Autonomous Vehicles" was published in 2022. Journal: Comput Intell Neurosci.

**Figure 2:** Proposed privacy-preserved intelligent IMS. Here, the identity features (*ID*s) are as follows: real face ID (*ID*_*R*_), anonymized face ID (*ID*_*A*_), ID of the occupant that caused an abnormal situation (*ID*_*A_AS*_), and suspect face ID during the investigation (*ID*_*inv*_).

**Figure 3:** Illustration of 128D facial identity feature vector generation (from the occupant's face image). Image shown is taken from our in-cabin monitoring database. The numerical values in the yellow, red, green, and blue colored boxes are representing respective passengers' (128, 1)-dimensional facial identity feature vectors (*ID*).

**Figure 4:** Source image generation using AI-generated faces with the best matching technique.

**Figure 5:** Set of virtual human faces (AI-generated faces). These virtual human faces are obtained from Generated Photos. It provides AI-generated images that are free from any copyrights, distribution rights, and infringement claims (source: Generated Photos (https://generated.photos/)).

**Figure 6:** We have chosen single and multiple faces in the input images in different scenarios: single face (only male or only female), multiple faces (only male), multiple faces (only female), and multiple faces (both male and female). Here, the target (occupant) faces are indexed from F1 to F23, and considered source faces (both male and female) are indexed from S1 to S4.

**Figure 7:** Facial anonymization with reenactment. F1 to F23: original images. A1 to A23: corresponding anonymized images considering appropriate source faces.

**Figure 8:** Snippets of our database showing vandalism inside the vehicle cabin. The original image under normal and irregular situations is in row R1, and the corresponding anonymized images are shown in row R2. The occupants are numbered from left to right clockwise (O1, O2, O3, and O4). Scene #1: O3 shakes shoulder of O4; scene #2: O3 tries to slap O4; scene #3 O3 shakes head of O4; and scene #4: O3 chokes neck of O4. Green box: concerned person and red box: in-cabin vandalism.

**Figure 9:** Other pictures of the occupants during investigation for matching. The numbering is the same as those in the in-cabin images from left to right (O1′', O2′', O3′', and O4′').

The article "Privacy-Preserved In-Cabin Monitoring System for Autonomous Vehicles" was published in 2022. Journal: Comput Intell Neurosci.

**Algorithm 1:** Algorithm for obtaining the ID of a person involved in an abnormal situation.

**Algorithm 2:** Algorithm for evidence of the person involved in the abnormal situation.

**Table 1:** Similarities between the source and target faces.

Scenario		Target (occupants^†^)	Similarity measure (using Euclidean distance)			
			S1	S2	S3	S4
Single face	Male	F1	0.91489481	0.80287961	0.89433056	**0.74069120**
	Female	F2	0.78818484	0.81636149	**0.68592050**	0.76422129
Multiple face	Male	F3	0.91414391	0.88400388	0.87615788	**0.83486502**
		F4	0.79685733	**0.71862379**	0.93450242	0.75311709
	Male	F5	0.91205174	0.82094296	0.87266242	**0.78036428**
		F6	0.81236709	0.80381698	0.93859941	**0.67143296**
	Female	F7	0.81097788	0.82709409	**0.71891988**	0.86480495
		F8	0.85947196	0.78512872	**0.77978978**	0.90500906
	Both	F9	0.89428390	0.83158545	0.88401185	**0.80949051**
	Both	F10	0.84977716	0.90480697	**0.71174311**	0.94153902
	Both	F11	0.65831500	**0.52838455**	0.95610671	0.88142326
	Both	F12	**0.38916649**	0.45361382	0.89109294	0.88496564
	Both	F13	0.79624321	0.80097813	0.88202307	**0.71975099**
	Both	F14	**0.63660264**	0.67343593	0.88004248	0.96042187
	Both	F15	0.84524707	0.89008615	**0.77500429**	0.86828727
	Both	F16	0.74547080	0.77676084	0.93155677	**0.73583944**
	Both	F17	0.79179192	0.80390987	**0.73040828**	0.88839209
	Both	F18	0.78950908	0.79986798	**0.72049968**	0.94658813
	Both	F19	0.90007099	0.85322199	0.99829307	**0.85322199**
	Both	F20	**0.40197132**	0.63806865	0.83032199	0.88047087
	Both	F21	**0.46230089**	0.53098278	0.85879277	0.86241199
	Both	F22	**0.48055832**	0.54356384	0.83216505	0.81304802
	Both	F23	0.55751665	**0.45767183**	0.90473598	0.78517239

^†^The occupants are numbered from left to right clockwise.

**Table 2:** Identity feature matching between *ID*_*A_IS*_#3 at the data center and other stored *ID*s of the occupants in the cloud for different scenarios.

Scene	Similarity measure (in Euclidean distance)			
	*ID*_*A*_#1	*ID*_*A*_#2	*ID*_*A*_#3	*ID*_*A*_#4
Scene #1	0.52893346	0.78363186	**0.35424358**	0.42124692
Scene #2	0.45234707	0.79687774	**0.35880417**	0.40963131
Scene #3	0.49863882	0.77615540	**0.41716736**	0.44500655
Scene #4	0.74701755	0.5816643	**0.53716927**	0.73605501

Detail description of scenes (scenes #1–#4) is mentioned in Section 3.2.

**Table 3:** Identity feature matching between the occupants' *ID*s extracted during the investigation and their *ID*s extracted from in-cabin images.

Occupant's *ID* (in-cabin)	Occupant's *ID*s were extracted during an investigation			
	*ID*_*O1*_'	*ID*_*O2*_'	*ID*_*O3*_'	*ID*_*O4*_'
*ID*_*O1*_	**0.48432609**	0.79061829	0.72076523	0.69776956
*ID*_*O2*_	0.75859866	**0.66392154**	0.79348079	0.72322158
*ID*_*O3*_	0.52265982	0.77696899	**0.36226176**	0.47469558
*ID*_*O4*_	0.64218059	0.81529880	0.52173335	**0.42871777**

The article "Privacy-Preserved In-Cabin Monitoring System for Autonomous Vehicles" was published in 2022. Journal: Comput Intell Neurosci.

**Table 4:** Identity feature matching between *ID*_*R*_ stored in the cloud with other occupant's *ID*s extracted from the in-cabin of the vehicle.

*ID* (person involved)	*IDs of the occupants (In-cabin)*			
	*ID*_*O1*_	*ID*_*O2*_	*ID*_*O3*_	*ID*_*O4*_
*ID*_*R*_	0.62511349	0.75967812	**0**	0.52087737

## Data Availability

The image data used to support the findings of this study are included in this paper.

## References

[1] Vennam P., Pramod T. C., Thippeswamy B. M., Kim Y.-G., Pavan Kumar B. N. (2021). Attacks and preventive measures on video surveillance systems: a review. *Applied Sciences*.

[2] Janai J., Güney F., Behl A., Geiger A. (2020). Computer vision for autonomous vehicles: problems, datasets and state of the art. *Foundations and Trends in Computer Graphics and Vision*.

[3] (February 2021). SAE international releases updated visual chart for its “levels of driving automation” standard for self-driving vehicles. https://www.sae.org/news/press-room/2018/12/sae-international-releases-updated-visual-chart-for-its-%E2%80%9Clevels-of-driving-automation%E2%80%9D-standard-for-self-driving-vehicles.

[4] (25 February 2021). Automated vehicles for safety. https://www.nhtsa.gov/technology-innovation/automated-vehicles-safety.

[5] Mishra A., Kim J., Kim D., Cha J., Kim S. An intelligent in-cabin monitoring system in fully autonomous vehicles.

[6] (February 2021). UK’s facial recognition technology ‘breaches privacy rights. https://www.theguardian.com/technology/2020/jun/23/uks-facial-recognition-technology-breaches-privacy-rights.

[7] (February 2021). Facial recognition technology privacy and accuracy issues related to commercial uses. https://www.gao.gov/assets/710/708045.pdf.

[8] (February 2021). Facial recognition technology fundamental rights considerations in the context of law enforcement. https://fra.europa.eu/en/publication/2019/facial-recognition-technology-fundamental-rights-considerations-context-law.

[9] Climent-Pérez P., Florez-Revuelta F. (2021). Protection of visual privacy in videos acquired with RGB cameras for active and assisted living applications. *Multimedia Tools and Applications*.

[10] Bignami F. (2020). *Schrems II: The Right to Privacy and the New Illiberalism*.

[11] Dushi D. (2020). *The Use of Facial Recognition Technology in EU Law Enforcement: Fundamental Rights Implications*.

[12] Mekrani A. (2020). *The Future of Facial Recognition in Relation to Privacy,” Master Thesis*.

[13] Naranjo D. (2020). *Your Face Rings a bell: How Facial Recognition Poses a Threat for Human Rights*.

The article "Privacy-Preserved In-Cabin Monitoring System for Autonomous Vehicles" was published in 2022. Journal: Comput Intell Neurosci.

[14] (February 2021). How facial recognition technology threatens basic privacy rights. https://www.computerweekly.com/feature/How-facial-recognition-technology-threatens-basic-privacy-rights.

[15] Doktor M. (2021). Facial recognition and the fourth amendment in the wake of carpenter v. United States. *University of Cincinnati Law Review*.

[16] Daly A. (2017). Privacy in automation: an appraisal of the emerging Australian approach. *Computer Law & Security Review*.

[17] Smith M., Miller S. (2021). The ethical application of biometric facial recognition technology. *AI & Society*.

[18] Van Noorden R. (2020). The ethical questions that haunt facial-recognition research. *Nature*.

[19] (July 2021). Facial-recognition research needs an ethical reckoning. https://www.nature.com/articles/d41586-020-03256-7.

[20] Rooijen A. V., Bouma H., Pruim R., Baan J., Uijens W., Mil J. V. Anonymized person re-identification in surveillance cameras. http://toc.proceedings.com/56397webtoc.pdf.

[21] Rong Y., Han C., Hellert C., Loyal A., Kasneci E. (2021). Artificial intelligence methods in in-cabin use cases: a survey. http://arxiv.org/abs/2101.02082.

[22] Marcondes F. S., Durães D., Gonçalves F., Fonseca J., Machado J., Novais P. (2021). In-vehicle violence detection in carpooling: a brief survey towards a general surveillance system. *Advances in Intelligent Systems and Computing*.

[23] Bell J. L., Taylor M. A., Chen G.-X., Kirk R. D., Leatherman E. R. (2017). Evaluation of an in-vehicle monitoring system (IVMS) to reduce risky driving behaviors in commercial drivers: comparison of in-cab warning lights and supervisory coaching with videos of driving behavior. *Journal of Safety Research*.

[24] Szawarski H., Le J., Rao M. K. (April 2019). Monitoring a vehicle cabin.

[25] Song X. (February 2019). Safety and clean vehicle monitoring system.

[26] Taeihagh A., Lim H. S. M. (2019). Governing autonomous vehicles: emerging responses for safety, liability, privacy, cybersecurity, and industry risks. *Transport Reviews*.

[27] Glancy D. J. (2012). Privacy in autonomous vehicles. *Santa Clara University School of Law*.

[28] Collingwood L. (2017). Privacy implications and liability issues of autonomous vehicles. *Information and Communications Technology Law*.

[29] Lim H. S. M., Taeihagh A. (2017). Autonomous vehicles for smart and sustainable cities: an in-depth exploration of privacy and cybersecurity implications. *Energies*.

[30] Rocher L., Hendrickx J. M., de Montjoye Y. A. (2019). Estimating the success of re-identifications in incomplete datasets using generative models. *Nature Communications*.

The article "Privacy-Preserved In-Cabin Monitoring System for Autonomous Vehicles" was published in 2022. Journal: Comput Intell Neurosci.

[31] Mishra A., Cha J., Kim S. HCI based in-cabin monitoring system for irregular situations with occupants facial anonymization.

[32] Nakamura T., Sakuma Y., Nishi H. (2021). Face-image anonymization as an application of multidimensional data k-anonymizer. *International Journal of Networking and Computing*.

[33] Moschoglou S., Ploumpis S., Nicolaou M. A., Papaioannou A., Zafeiriou S. (2020). 3DFaceGAN: adversarial nets for 3D face representation, generation, and translation. *International Journal of Computer Vision*.

[34] Hukkelås H., Mester R., Lindseth F. DeepPrivacy: a generative adversarial network for face anonymization.

[35] Dietlmeier J., Antony J., McGuinness K., O Connor N. E. (2020). How important are faces for person re-identification?. http://arxiv.org/abs/2010.06307.

[36] Sun Q., Tewari A., Xu W., Fritz M., Theobalt C., Schiele B. A hybrid model for identity obfuscation by face replacement.

[37] Blanz V., Scherbaum K., Vetter T., Seidel H.-P. (2004). Exchanging faces in images. *Computer Graphics Forum*.

[38] Bitouk D., Kumar N., Dhillon S., Belhumeur P., Nayar S. K. (2008). Face swapping. *ACM Transactions on Graphics*.

[39] Zhang Y., Zheng L., Thing V. L. Automated face swapping and its detection.

[40] Nirkin Y., Masi I., Tuan A. T., Hassner T., Medioni G. On face segmentation, face swapping, and face perception.

[41] Kim T., Yang J. (2020). Selective feature anonymization for privacy-preserving image data publishing. *Electronics*.

[42] Natsume R., Yatagawa T., Morishima S. (2018). RSGAN: face swapping and editing using face and hair representation in latent spaces. http://arxiv.org/abs/1804.03447.

[43] Korshunov P., Marcel S., Fakes D. (2018). A new threat to face recognition? Assessment and detection. http://arxiv.org/abs/1812.08685.

[44] Natsume R., Yatagawa T., Morishima S. (2019). FSNet: an identity-aware generative model for image-based face swapping. *Computer Vision - ACCV 2018*.

[45] Bailer W. Face swapping for solving collateral privacy issues in multimedia analytics.

[46] Nirkin Y., Keller Y., Hassner T. FSGAN: subject agnostic face swapping and re-enactment.

[47] Naruniec J., Helminger L., Schroers C., Weber R. M. (2020). High -resolution neural face swapping for visual effects. *Computer Graphics Forum*.

[48] Jain A. K., Li S. Z. (2011). *Handbook of Face Recognition*.

[49] Huang T., Xiong Z., Zhang Z. (2005). *Face Recognition Applications, Handbook of Face Recognition*.

[50] Parmar D. N., Mehta B. B. (2014). Face recognition methods & applications. http://arxiv.org/abs/1403.0485.

[51] Adjabi I., Ouahabi A., Benzaoui A., Taleb-Ahmed A. (2020). Past, present, and future of face recognition: a review. *Electronics*.

The article "Privacy-Preserved In-Cabin Monitoring System for Autonomous Vehicles" was published in 2022. Journal: Comput Intell Neurosci.

[52] Kortli Y., Jridi M., Al Falou A., Atri M. (2020). Face recognition systems: a Survey. *Sensors*.

[53] Turk M., Pentland A. (1991). Eigenfaces for recognition. *Journal of Cognitive Neuroscience*.

[54] Belhumeur P. N., Hespanha J. P., Kriegman D. J. (1997). Eigenfaces vs. Fisherfaces: recognition using class specific linear projection. *IEEE Transactions on Pattern Analysis and Machine Intelligence*.

[55] Taigman Y., Yang M., Ranzato M., Wolf L. DeepFace: closing the gap to human-level performance in face verification.

[56] Sun Y., Wang X., Tang X. Deep learning face representation from predicting 10,000 classes.

[57] Sun Y., Chen Y., Wang X., Tang X. Deep learning face representation by joint identification-verification.

[58] Sun Y., Wang X., Tang X. Deeply learned face representations are sparse, selective, and robust.

[59] Sun Y., Liang D., Wang X., Tang X. (2015). DeepID3: face recognition with very deep neural networks. http://arxiv.org/abs/1502.00873v1.

[60] Wang M., Deng W. (2021). Deep face recognition: a survey. *Neurocomputing*.

[61] Erkin Z., Franz M., Guajardo J., Katzenbeisser S., Lagendijk I., Toft T. Privacy-preserving face recognition.

[62] Roussi A. (2020). Resisting the rise of facial recognition. *Nature*.

[63] Luo H., Gu Y., Liao X., Lai S., Jiang W. Bag of tricks and a strong baseline for deep person re-identification.

[64] He K., Zhang X., Ren S., Sun J. Deep residual learning for image recognition.

[65] Schroff F., Kalenichenko D., Philbin J. FaceNet: a unified embedding for face recognition and clustering.

[66] King D. E. (2009). Dlib-ml: a machine learning toolkit. *Journal of Machine Learning Research*.

[67] Kim J., Cha J., Kim S. (2020). Hands-free user interface for VR headsets based on in situ facial gesture sensing. *Sensors*.

[68] Cha J., Kim J., Kim S. (2019). Hands-free user interface for AR/VR devices exploiting wearer’s facial gestures using unsupervised deep learning. *Sensors*.

